The article "Clinical Evaluation of Pinggan Yiqi Yangshen Recipe Combined with Labetalol Hydrochloride and Magnesium Sulfate in the Treatment of PIH" was published in 2021. Journal: Evid Based Complement Alternat Med.

# Clinical Evaluation of Pinggan Yiqi Yangshen Recipe Combined with Labetalol Hydrochloride and Magnesium Sulfate in the Treatment of PIH

**DOI:** 10.1155/2021/3135043

**Published:** 2021-10-28

**Authors:** Ping Li, Jie Zhao, Peipei Gao, Hongcui Qu

**Affiliations:** ^1^Health Education Department, Zhangqiu Maternity and Child Care Hospital, Jinan 250200, China; ^2^Outpatient Department, Zhangqiu Maternity and Child Care Hospital, Jinan 250200, China; ^3^Comprehensive Ward, Zhangqiu Maternity and Child Care Hospital, Jinan 250200, China; ^4^Outpatient Operating Room, Zhangqiu Maternity and Child Care Hospital, Jinan 250200, China

## Abstract

**Background:**

To observe the clinical effect of Pinggan Yiqi Yangshen recipe combined with labetalol hydrochloride and magnesium sulfate in the treatment of pregnancy-induced hypertension (PIH).

**Methods:**

A total of 126 patients with PIH diagnosed in our hospital from January 2016 to May 2018 were randomly divided into the control group and the experimental group, with 63 cases in each group. The control group was treated with labetalol combined with magnesium sulfate. On the basis of the control group, the experimental group was treated with Pinggan Yiqi Yangshen recipe. Clinical efficacy, blood pressure, renal function, and biochemical indexes were compared between the two groups. Moreover, pregnancy outcomes and adverse reactions were compared between the two groups.

**Results:**

After treatment, the total effective rate in the experimental group was higher than in the control group. Blood pressure and mean arterial pressure in the experimental group were more significantly downregulated than the control group. Renal function indexes and biochemical indexes in the experimental group were more significant than those in the control group. The incidence of cesarean section, preterm birth, and abnormal fetal heart rate in the experimental group was significantly lower than that in the control group. There was no difference in the incidence of fetal distress, postpartum hemorrhage, neonatal asphyxia, and adverse reactions between the two groups.

**Conclusion:**

Pinggan Yiqi Yangshen recipe combined with labetalol hydrochloride and magnesium sulfate can effectively reduce the blood pressure of patients with PIH, help patients to return to normal levels of biochemical indexes and renal function indexes, and improve pregnancy outcomes with high safety, which is worthy of further promotion and application in clinical practice.

## 1. Introduction

Pregnancy-induced hypertension (PIH) is a disease that occurs more frequently in pregnant women. PIH usually refers to a pregnancy complication with hypertension, nausea, vomiting, edema, and proteinuria as the main clinical symptoms after 20 weeks of pregnancy [1, 2]. If not treated timely, patients will suffer from convulsion, coma, heart failure, kidney failure, and other serious conditions and can also cause fetal distress, premature delivery, and even death. PIH seriously threatens the life safety of the mother and child and is one of the main causes of maternal death at present [3]. In recent years, the incidence of PIH has been increasing year by year [4], which has aroused great attention from doctors and patients. Clinically, western medicine is mainly used to treat patients with PIH, among which magnesium sulfate and labetalol hydrochloride are the most common [4, 5]. However, long-term use may lead to some adverse reactions in patients, such as weakened knee reflex and muscle weakness [6]. At present, western medicine combined with traditional Chinese medicine has been gradually used to treat PIH, and its advantages have been reported in clinical practice. It can not only play the advantage of the rapid therapeutic effect of western medicine but also reflect the characteristics of the overall adjustment and treatment of both symptoms and root causes of traditional Chinese medicine [7, 8].

The article "Clinical Evaluation of Pinggan Yiqi Yangshen Recipe Combined with Labetalol Hydrochloride and Magnesium Sulfate in the Treatment of PIH" was published in 2021. Journal: Evid Based Complement Alternat Med.

In this study, Pinggan Yiqi Yangshen recipe was used in combination with labetalol hydrochloride and magnesium sulfate to treat PIH in order to observe its clinical effect on PIH and the occurrence of adverse outcomes during pregnancy.

## 2. Materials and Methods

### 2.1. General Information

A total of 126 patients with PIH admitted to Zhangqiu Maternity and Child Care Hospital from January 2016 to May 2018 were randomly divided into the experimental group (63 cases) and control group (63 cases). There was no significant difference in general data between the two groups (*P* > 0.05, Table 1). The inclusion criteria were as follows: all patients met the diagnostic criteria of PIH in “Obstetrics & Gynecology” [9]; all patients were singleton pregnancies; all patients were treated for the first time. The exclusion criteria were as follows: patients with serious heart, brain, kidney, liver, and other important viscera-related diseases; patients who are allergic to the treatment drugs in this study; patients who do not cooperate with the researcher. This study was approved by the ethics committee of Zhangqiu Maternity and Child Care Hospital, and all patients signed informed consent.

### 2.2. The Treatment

The patients in both groups were treated with 0.25–5 g methyldopa (H11020968, China Resources Shuanghe Pharmaceutical Co., Ltd.), twice a day. The control group was treated with basic treatment combined with labetalol hydrochloride and magnesium sulfate. The usage and dosage of labetalol hydrochloride were as follows: the patients received an intravenous infusion of 50 mg labetalol hydrochloride (H32026120, Jiangsu Desano Pharmaceutical Co., Ltd.) dissolved in 250 ml of 5% glucose solution at 2 mg/min, once a day, for 7 days. Severe patients were given 30 ml 10% glucose solution containing 25 mg labetalol hydrochloride by an intravenous drip. The usage and dosage of magnesium sulfate were as follows: the patients received an intravenous infusion of 60 ml magnesium sulfate injection (national drug approval H33021961, Hangzhou Minsheng Pharmaceutical Co., Ltd.) dissolved in 500 ml 5% glucose injection at 1-2 g/h, once a day, for 7 days. The experimental group was added with Pinggan Yiqi Yangshen recipe on the basis of the control group. The prescription of Pinggan Yiqi Yangshen recipe was as follows: 15 g *Eucommia ulmoides*, 10 g *Uncaria rhynchophylla*, 30 g *Astragali Radix*, 20 g *Semen Cassiae*, 20 g *Chrysanthemum morifolium*, 15 g *Poria cocos*, 15 g *Atractylodes macrocephala*, 15 g *Bupleurum chinense*, 20 g *Curcumae Radix*, 30 g *Radix Codonopsis*, 10 g *Rhizoma Alismatis*, 6 g *Pinelliae Rhizoma*, 20 g *Angelica*, 15 g *Angelica dahurica*, 10 g *Gardenia jasminoides*, 10 g *Citri Reticulatae Pericarpium*, 10 g *Cyperus rotundus*, 10 g *Paeoniae Alba Radix*, 5 g *Cortex Phellodendri*, 15 g donkey-hide gelatin, and 15 g *Herba Taxilli* were decocted with water every morning and evening for 7 days, one course of treatment for light patients and two courses of treatment for severe patients.

The article "Clinical Evaluation of Pinggan Yiqi Yangshen Recipe Combined with Labetalol Hydrochloride and Magnesium Sulfate in the Treatment of PIH" was published in 2021. Journal: Evid Based Complement Alternat Med.

### 2.3. Observation Indexes

The clinical effect of patients in two groups after treatment was observed. The criteria were as follows: (1) special effect: the patient's symptoms and signs were disappeared, the systolic blood pressure (SBP) was decreased >30 mmHg, the diastolic blood pressure (DBP) was decreased >20 mmHg, the blood pressure was normal, and 24 h urine protein (Upro) was decreased; (2) valid effect: the patients' symptoms and signs were disappeared or improved, SBP was decreased <10 mmHg, DBP was decreased <120 mmHg, blood pressure was basically normal, and Upro was decreased; (3) invalid effect: the patients' symptoms, signs, blood pressure, and Upro were not changed or worse. Total effective rate = (special + valid)/total cases.

The improvement of blood pressure and mean arterial pressure before and after treatment was observed. The biochemical indexes of the two groups were detected. Biuret colorimetry (BT 2000 Plus Biochemical Analyzer, Italy BT) was used to detect the level of 24 h Upro. The level of superoxide dismutase (SOD) was measured by the xanthine oxidase assay (Xanthine Oxidase Test Kit, Shenzhen Zike Biotechnology Co., Ltd.). The plasma nitric oxide (NO) level was determined by nitric acid reductase (Nitric Oxide Test Kit, Shanghai Yisen Biological Technology Co., Ltd.). The level of malondialdehyde (MDA) was determined by the thiobarbituric acid method (Shanghai Mingbo Biological Technology Co., Ltd.). The plasma endothelin-1 (ET-1) level was determined by the radioimmunoassay (Shanghai Hengyuan Biological Technology Co., Ltd.). Renal function indexes were detected in both groups. The normal range of blood urea nitrogen (BUN) was 3.2–7.1 mmol/L; serum creatinine (Cr) was 70–106 *μ*mol/L; serum uric acid (UA) was 89–357 *μ*mol/L; serum urea (SU) was 1.78–7.14 mmol/L. The adverse reactions and maternal and infant outcomes of the two groups were observed.

The article "Clinical Evaluation of Pinggan Yiqi Yangshen Recipe Combined with Labetalol Hydrochloride and Magnesium Sulfate in the Treatment of PIH" was published in 2021. Journal: Evid Based Complement Alternat Med.

### 2.4. Statistical Analysis

SPSS 22.0 software was used to analyze the data. The measurement data was expressed as $\bar{x}+s$, and the counting data were expressed as *n* (%) and analyzed by *X*^2^ test. *P* < 0.05 was considered statistically significant.

## 3. Results

### 3.1. Comparison of Clinical Efficacy between the Two Groups

The total effective rate of the experimental group was 93.65%, and that of the control group was 71.43%. The clinical efficacy of the treatment group was significantly higher than that of the control group (*X*^2^ = 16.211, *P* < 0.01, Table 2).

### 3.2. Comparison of Renal Function Indexes and Biochemical Indexes in Two Groups

There was no significant difference in renal function and biochemical indexes between the two groups before treatment. After treatment, renal function indexes and biochemical indexes in both groups decreased compared with those before treatment, and the reduction in the experimental group was more significant than that in the control group (*P* < 0.01, Tables 3 and 4).

### 3.3. Comparison of Blood Pressure and Mean Arterial Pressure in Two Groups

Before treatment, there was no significant difference in blood pressure between the experimental group and control group (*P* > 0.05). After treatment, SBP was 127.63 ± 11.45 mmHg, DBP was 78.34 ± 15.71 mmHg, and MAP was 101.66 ± 6.23 mmHg. In the control group, SBP was 151.32 ± 13.16 mmHg, DBP was 90.57 ± 16.63 mmHg, and MAP was 121.37 ± 7.54 mmHg. SBP, DBP, and MAP in both groups were lower than before treatment (*P* < 0.05), and the experimental group was more significantly decreased than the control group (*P* < 0.05, Figures 1 and 2).

### 3.4. Comparison of the Incidence of Adverse Reactions and Pregnancy Outcomes between the Two Groups

After treatment, the incidence of cesarean section, preterm birth, and abnormal fetal heart rate in the experimental group was significantly lower than that in the control group (*P* < 0.05). There was no significant difference in the incidence of fetal distress, postpartum hemorrhage, and neonatal asphyxia between the two groups (*P* > 0.05). There was no significant difference in the incidence of adverse reactions between the two groups (*P* > 0.05, Tables 5 and 6).

The article "Clinical Evaluation of Pinggan Yiqi Yangshen Recipe Combined with Labetalol Hydrochloride and Magnesium Sulfate in the Treatment of PIH" was published in 2021. Journal: Evid Based Complement Alternat Med.

## 4. Discussion

PIH is caused by many factors, such as family genetic history, age, obesity, and hypertension. At the same time, insufficient nutritional intake and recurrent mood fluctuations during pregnancy can also lead to the occurrence of PIH [10, 11]. The main clinical manifestations of PIH are abnormally elevated blood pressure, proteinuria, edema, etc., accompanied by dizziness, nausea, systemic small vessel spasm, and other clinical symptoms. Furthermore, due to the high blood pressure of patients, there will be insufficient blood supply in the uterus and placenta, which will affect the uptake of oxygen and nutrients in the uterus of the fetus and be prone to fetal intrauterine growth retardation and other phenomena. Severe cases are forced to terminate pregnancy or even die, which poses a serious threat to the life safety of pregnant women and fetus [12, 13]. Through effective intervention to control pregnant women's blood pressure, the occurrence of cardiovascular and cerebrovascular diseases can be avoided, which is of great significance to ensure the healthy development of the fetus and guarantee the life safety of pregnant women. At present, a single antihypertensive drug combined with lifestyle improvement is used to treat patients with PIH, but the treatment effect is not ideal [14]. Due to the poor physical quality of pregnant women, this situation is easy to cause adverse effects in the fetus [15, 16]. Labetalol hydrochloride is one of the antihypertensive drugs commonly used in the treatment of PIH, which can dilate blood vessels, reduce cardiac load and myocardial oxygen consumption, and increase cardiac output, so as to achieve the purpose of lowering blood pressure [17, 18]. Magnesium sulfate has the antagonistic effect of Ca^2+^ and is mainly used for anticonvulsion. It can reduce blood pressure by causing vascular dilation, further improve human microcirculation, and can be used for the treatment of hypertensive crisis [19, 20].

According to the traditional Chinese medicine system, due to the pregnancy of the fetus in the pregnant woman, all organs of the body cannot function normally, which will lead to the deficiency of the spleen and kidney yang deficiency, resulting in the disorder of water and moisture functions in the body [21]. Kidney yang deficiency leads to poor water flow in pregnant women and obstruction of fetal gas, resulting in the fetal and maternal deficiency of blood. Therefore, patients with PIH should tonify the kidney and qi [22]. In this paper, we study a TCM prescription of Pinggan Yiqi Yangshen recipe. Among them, *Astragali Radix* has the functions of tonifying qi, replenishing wei, and consolidating the exterior. *Radix Codonopsis* has the functions of tonifying qi and nourishing blood. *Cortex Phellodendri* and *Gardenia jasminoides* have the effects of clearing away heat, purging fire and dampness, and detoxification. *Paeoniae Alba Radix* and *Cyperus rotundus* have the effects of nourishing blood, softening the liver, and relieving pain. *Pinelliae Rhizoma* can dry wet and reduce phlegm. *Citri Reticulatae Pericarpium* has the function of regulating qi and dispelling phlegm. *Atractylodes macrocephala* and *Poria cocos* have the functions of moistening water, invigorating the spleen and stomach, and relieving the heart and placenta. *Curcumae Radix* and *Angelica* have the actions of supplementing blood, promoting blood circulation, and opening the meridians. *Chrysanthemum morifolium* and *Semen Cassiae* have the actions of calming liver wind. *Bupleurum chinense*, *Angelica dahurica*, and *Uncaria rhynchophylla* have the functions of relieving liver depression, calming liver wind, reinforcing qi, and elevating yang. *Rhizoma Alismatis* has the effect of inducing diuresis to alleviate edema. *Eucommia ulmoides*, donkey-hide gelatin, and *Herba Taxilli* have the actions of eliminating dampness, calming the liver, reinforcing the kidney, and preventing miscarriage. *Citri Reticulatae Pericarpium* has the functions of invigorating the spleen and regulating the stomach. The whole prescription can reinforce qi, strengthen the spleen, calm the liver, and reinforce the kidney [23–28]. Recent research has reported that *Atractylodes macrocephala* and *Poria cocos* can enhance human immunity [29, 30]. *Uncaria rhynchophylla* and *Eucommia ulmoides* have strong antihypertensive, sedative, spasmodic, and diuretic effects [31, 32]. *Chrysanthemum morifolium* extract solution can dilate blood vessels, reduce blood pressure, and reduce the cardiac output [33]. On the basis of western medicine use in hypertension, Chinese medicine can improve the possible adverse outcomes during pregnancy, improve human microcirculation, and can achieve the safe hypotension effect.

The article "Clinical Evaluation of Pinggan Yiqi Yangshen Recipe Combined with Labetalol Hydrochloride and Magnesium Sulfate in the Treatment of PIH" was published in 2021. Journal: Evid Based Complement Alternat Med.

This study showed that, after treatment, both groups had certain clinical treatment effects. Our results showed that the combination of traditional Chinese and western medicine could effectively reduce the blood pressure and improve the clinical symptoms of pregnancy hypertension. After treatment, the levels of BUN, UA, Cr, and SU in the experimental group were lower than those in the control group. We identified that this was closely related to the efficacy of *Astragali Radix, Herba Taxilli*, and *Eucommia ulmoides* in these prescriptions, such as nourishing qi and nourishing yuan, tonifying the kidney, calming the liver, and strengthening body resistance to eliminate pathogenic factors. Pinggan Yiqi Yangshen recipe can improve the renal blood circulation and increase the blood flow, and it significantly decreased the level of renal function indicators. After treatment, the incidences of cesarean section, premature birth, and abnormal fetal heart rate in the experimental group were significantly higher than those in the control group. However, there was no difference in the incidence of fetal distress, postpartum hemorrhage, and neonatal asphyxia between the two groups, which may be related to the small number of cases included. NO, an important diastolic factor produced by endothelial cells, is a new type of transport molecule with free radical properties with the effect of vascular dilation. SOD is an antioxidant enzyme to defend against the damage and destruction of oxygen free radical in metabolism and other life activities. MDA is a major metabolite reflecting lipid peroxidation in the body. The level of MDA in plasma can reflect the content of free radicals in tissues and the degree of lipid peroxidation damage. ET-1 exists in vascular endothelial cells and is one of the most vital vasoconstrictor factors. Plasma ET-1 is associated with hemodynamic changes during normal pregnancy. ET-1 showed no significant difference in the first and second trimester, but increased significantly in the third trimester, interacting with other vasoactive substances to regulate blood pressure and hemodynamic changes [34–37]. In this study, the levels of NO and SOD increased in both groups after treatment, and the experimental group was significantly higher than the control group. The levels of MDA, RT-1, and Upro in the experimental group were significantly lower than those in the control group. The results showed that the combination of integrated Chinese and western medicine is effective in treating PIH and can adjust the level of each index to the normal range.

In conclusion, Pinggan Yiqi Yangshen recipe combined with labetalol hydrochloride and magnesium sulfate can effectively improve the clinical symptoms of PIH patients, restore the damaged liver and kidney function, and improve the adverse outcomes during pregnancy in the mother and infant, which is worthy of further clinical promotion.

The article "Clinical Evaluation of Pinggan Yiqi Yangshen Recipe Combined with Labetalol Hydrochloride and Magnesium Sulfate in the Treatment of PIH" was published in 2021. Journal: Evid Based Complement Alternat Med.

## Figures and Tables

**Figure 1:** Comparison of the blood pressure between the two groups. (a) SBP in the experimental group was compared before and after treatment. (b) DBP in the experimental group was compared before and after treatment. (c) SBP in the control group was compared before and after treatment. (d) DBP in the control group was compared before and after treatment. ^*∗*^*P* < 0.05.

**Figure 2:** Comparison of the mean arterial blood pressure between the two groups. (a) MAP in the experimental group was compared before and after treatment. (b) MAP in the control group was compared before and after treatment. ^∗∗^*P* < 0.05.

**Table 1:** Comparison of general clinical data between the two groups.

Clinical parameters	Experimental group (*n* = 63)	Control group (*n* = 63)	*X* ^2^	*P* value
*Age (years)*				
≤32	37	40	0.301	0.584
>32	26	23		

*BMI (kg/m* ^*2*^)				
<18.5	6	8	0.725	0.696
18.5–24.9	45	46		
≥25	12	9		

*Gestational age (weeks)*				
<28	7	8	0.076	0.783
≥28	56	55		

*Parity*				
1	41	39	0.137	0.711
>1	22	24		

*Severity degree*				
Mild	8	9	0.469	0.791
Moderate	49	50		
Severe	6	4		

**Table 2:** Comparison of clinical efficacy between the two groups.

Group	*n*	Special effect	Valid effect	Invalid effect	Total effective rate
Experimental group	63	57.14% (36/63)	36.51% (23/63)	6.35% (4/63)	93.65% (59/63)
Control group	63	26.98% (17/63)	44.44% (28/63)	28.57% (18/63)	71.43% (45/63)
*X* ^2^					16.211
*P*					<0.01

**Table 3:** Comparison of biochemical indexes between two groups.

Group		NO (mmol/L)	SOD (U/ml)	24 h Upro (g)	ET-1 (ng/L)	MDA (nmol/L)
Experimental group	Before treatment	523.46 ± 72.84	63.21 ± 8.73	4.22 ± 1.14	93.56 ± 17.73	21.84 ± 6.12
	After treatment	971.43 ± 104.57^∗Δ^	124.37 ± 17.84^∗Δ^	1.25 ± 0.82^∗Δ^	48.65 ± 8.97^∗Δ^	10.76 ± 4.11^∗Δ^

Control group	Before treatment	525.71 ± 71.66	61.28 ± 8.16	4.18 ± 1.09	94.11 ± 18.06	21.63 ± 6.34
	After treatment	747.23 ± 79.47^*∗*^	92.64 ± 13.92^*∗*^	2.71 ± 0.94^*∗*^	73.24 ± 12.69^*∗*^	15.93 ± 4.45^*∗*^*s*

*X* ^2^		13.542	9.416	6.631	11.723	7.264

*P*		<0.01	<0.01	<0.01	<0.01	<0.01

Compared with the same group before treatment, ^*∗*^*P* < 0.01; compared with the control group after treatment, ^Δ^*P* < 0.01.

**Table 4:** Comparison of renal function indexes between two groups.

Group		Cr (*μ*mol/L)	SU (mmol/L)	BUN (mmol/L)	UA (*μ*mol/L)
Experimental group	Before treatment	123.47 ± 12.56	9.61 ± 1.67	8.97 ± 1.54	433.74 ± 52.67
	After treatment	83.96 ± 8.44^∗Δ^	4.54 ± 1.22^∗Δ^	4.26 ± 0.73^∗Δ^	236.71 ± 39.82^∗Δ^

Control group	Before treatment	122.76 ± 12.41	9.58 ± 1.72	8.83 ± 1.45	430.95 ± 53.74
	After treatment	99.42 ± 9.26^*∗*^	6.87 ± 1.53^*∗*^	5.64 ± 0.89^*∗*^	314.85 ± 42.36^*∗*^

*X* ^2^		11.124	6.173	8.265	13.814

*P*		<0.01	<0.01	<0.01	<0.01

Compared with the same group before treatment, ^*∗*^*P* < 0.01; compared with the control group after treatment, ^Δ^*P* < 0.01.

The article "Clinical Evaluation of Pinggan Yiqi Yangshen Recipe Combined with Labetalol Hydrochloride and Magnesium Sulfate in the Treatment of PIH" was published in 2021. Journal: Evid Based Complement Alternat Med.

**Table 5:** Comparison of the incidence of adverse reactions between two groups.

Group	*n*	Headaches	Nausea	Swelling	Vomiting	Muscle weakness
Experimental group	63	5	3	2	4	7
Control group	63	8	4	3	7	9
*X* ^2^		0.513	0.207	0.161	0.446	0.737
*P*		>0.05	>0.05	>0.05	>0.05	>0.05

**Table 6:** Comparison of pregnancy outcomes between the two groups after treatment.

Group	*n*	Caesarean section	Premature birth	Fetal distress	Postpartum hemorrhage	Abnormal fetal heart rate	Neonatal asphyxia
Experimental group	63	23	11	2	2	3	3
Control group	63	42	26	6	8	15	7
X^2^		5.623	4.216	0.451	0.782	7.667	0.486
*P*		<0.05	<0.05	>0.05	>0.05	<0.05	>0.05

## Data Availability

The data used to support the findings of this study are available from the corresponding author upon request.
